# Endovascular Intervention in a Narrowing Vessel of the Left Vertebral Artery with Bilateral Common Carotid Artery Occlusion and Aneurysm Rupture and Hemorrhage in the V4 Segment of the Right Vertebral Artery

**DOI:** 10.1155/2022/3279090

**Published:** 2022-05-19

**Authors:** Yang Feng, Han Peng, Xin Xiang, Xi Zeng, Bin Sun, Hongyi Lin, Xiaofeng Wang, Hua Yang

**Affiliations:** ^1^Guizhou Medical University, Guiyang 550000, China; ^2^Department of Neurosurgery, Affiliated Hospital of Guizhou Medical University, Guiyang 550000, China; ^3^Shandong First Medical University, Tai'an 250000, China

## Abstract

In this study, a case of bilateral common carotid artery occlusion and aneurysm in the V4 segment of the right vertebral artery with constriction of the left vertebral artery is presented. By improving digital subtraction angiography, an elderly female patient with subarachnoid haemorrhage (SAH) was diagnosed with a V4 segment of right vertebral artery aneurysm, a microaneurysm at the beginning of basilar aneurysms, bilateral common carotid artery occlusion, and narrowing vessel of left vertebral artery (DSA). Through the compensation of the basilar artery, the bilateral vertebral arteries provide intracranial and extracranial blood. Because the vertebral artery is narrowed, the right vertebral artery has priority in intracranial and extracranial blood delivery. Many members of the patient's immediate family have vasculitis, which has yet to be proven by appropriate laboratory testing but is thought to be the major cause of big artery occlusion. After cerebral angiography, the major source of this subarachnoid haemorrhage was determined to be a V4 segment of right vertebral artery aneurysm. Endovascular stent-assisted coil embolization was used to treat a V4 section of the right vertebral artery aneurysm. Because the basilar aneurysm was distal to the artery, interventional embolization was difficult to do, and it was not the major cause of the subarachnoid haemorrhage, the patient was advised to have follow-up surveillance, and she recovered well following the procedure. The combination of endovascular intervention of bilateral common carotid artery blockage and V4 segment of right vertebral artery aneurysm yielded excellent clinical outcomes in this instance. Endovascular treatment of a bilateral common carotid artery blockage paired with a V4 segment of a right vertebral artery aneurysm yielded excellent clinical outcomes in this patient, although long-term follow-up is necessary.

## 1. Introduction

The existence of a thin contralateral vertebral artery with bilateral common carotid artery blockage and vertebral artery aneurysm is extremely unusual. When the common carotid artery is blocked bilaterally, the whole cerebral blood supply is dependent on the supply of vertebrobasilar arteries, and owing to aberrant haemodynamics, the vessels and their branches along the pathway are subjected to excessively high pressure, resulting in aneurysms. At the same time, aneurysms are easily ruptured and bleed under the effect of numerous stimuli. Aneurysms of this kind have a significant mortality rate [1]. As a result, such aneurysms should be carefully managed to avoid rebleeding and life-threatening complications [2]. Because of the reverse flow from the external to the internal carotid artery and the cerebral compensation of the Willis vascular ring, patients with chronic bilateral common carotid artery blockage (chronic on at least one side) are less likely to appear with particular clinical symptoms [3]. Since its initial publication in 1991, intravascular interventional treatment has been frequently employed in clinic.

It has the features of a little injury and precise location. The limitations of partial craniotomy and clipping are alleviated by intravascular interventional treatment. Furthermore, it is the therapy of choice for the majority of cerebrovascular disorders [4]. The burst aneurysm was embolized by endovascular stent-assisted coil embolization in a case of bilateral common carotid artery blockage and V4 segment of right vertebral artery aneurysm with a narrow left vertebral artery. Although a good prognosis has been attained, long-term monitoring is still required.

In this study, a case of bilateral common carotid artery occlusion and aneurysm in the V4 segment of the right vertebral artery with constriction of the left vertebral artery is presented. To verify the claim, experimental observations were carried out by extensively examining patients with these diseases and symptoms in the hospital. A good and effective prognosis has been attained through those experiments, but long-term monitoring and extensions are still applicable and required.

The rest of the study is organized as given below.

In Section 2, the proposed treatment methodology is presented where a case study is thoroughly investigated and reported. In Section 3, treatment procedure and methodology is described in detail. Results and observation of the experiments are reported in Section 3 along with both textual and graphical representations. Finally, concluding remarks are given.

## 2. Proposed Treatment Methodology

The patient is a 53-year-old woman. She was brought to the hospital for 14 hours due to a rapid onset of headache, nausea, and vomiting. She experienced a rapid onset of headache with no obvious reason, which was a strong, diffuse, and dissipating pain that radiated to the neck and intensified in paroxysms and which did not improve with rest. At the same time, there were nausea and vomiting symptoms, including nonprojectile vomiting of stomach content. The patient was sent to another hospital's emergency neurology department. The DSA revealed “(1) V4 segment of right vertebral artery aneurysm, (2) aneurysm of the traffic segment of the left internal carotid artery, (3) bilateral common carotid artery blockage, and (4) slender left vertebral artery,” according to the CT scan. For additional treatment, she was admitted to our hospital. Cervical tonicity, three transverse fingers, limb muscle strength grade IV, normal muscle tone, drowsy, partially cooperative, and bilateral pupils were equal in size and about 2.5 mm in diameter, bilateral direct and indirect light reflexes were sensitive, bilateral direct and indirect light reflexes were sensitive, bilateral direct and indirect light reflexes were sensitive, cervical tonicity, three transverse fingers, limb muscle strength grade IV, normal muscle tone Meningeal GCS score: 13, Babinski's sign (−), Chaddock's sign (−), Oppenheim's sign (−), and Gordon's sign (−). Hunt-Hess score: 3; enhanced Fisher's scale: III; eyes open 3, speech 4, and movement 6; Hunt-Hess score: 3; improved Fisher's scale: III. She had previously been hospitalised in another hospital 30 years ago for rapid onset of awareness and was diagnosed with bilateral common carotid artery blockage, but neither the patient nor her relatives could recollect the specific diagnosis. Furthermore, she had TB 28 years ago, which was successfully treated with anti-tuberculosis medicine. Several members of her family have a history of vasculitis. The patient was brought to the hospital for a follow-up cranial CT scan: (1) a shuttle-shaped hyperdensity shadow in the right cerebellar hemisphere (size 11 mm 8 mm), with consideration of a haematoma; (2) subarachnoid haemorrhage, bilateral blood accumulation in the lateral ventricles, third ventricle, and fourth ventricle, and fluid accumulation in the supratentorial ventricles; (3) subarachnoid haemorrhage, bilateral blood accumulation in the lateral ventricles and third ventricle. The following are the admission diagnoses: (1) spontaneous subarachnoid haemorrhage and rupture into the ventricles; (2) spontaneous subarachnoid haemorrhage and rupture into the ventricles. After admission, the patient received critical care, haemostasis, seizure prevention, acid suppression, and gastrointestinal protection, prevention of vasospasm, and intravenous rehydration. All of the P-ANCA, C-ANCA, ANCA-MPO, ANCA-PR3, and ACA tests were negative. A full brain angiography was conducted under general anaesthetic after getting approval from the patient's relatives.

## 3. Procedure: Methodology

After general anaesthesia had taken effect, the surgical area was disinfected and sterile towels and sheets were laid out. The right femoral artery was punctured with Seldinger' method and after successful placement of the 8F arterial catheter sheath, heparin saline was injected. The 5 F Pigtail catheter was guided by a guide wire to the aortic arch for angiography. Then, bilateral common carotid artery occlusion was seen, the left vertebral artery was slender, and the right vertebral artery was significantly thickened. The 5 F Pigtail catheter was subsequently placed into the opening of the vertebral artery, with a tortuous vascular pathway and multiple collateral circulation seen to be established around it, and consideration was given to compensating for the rest of the intracranial blood supply via the posterior cerebral circulation (Figures 1(a) and 1(b)). A narrow carotid aneurysm was seen in the V4 segment of the right vertebral artery, with a neck of approximately 2.2 mm and a body of approximately 7.9 mm ∗ 7.5 mm (Figure 2: Figure 2(a) is frontal view; Figure 2(b) is lateral view), and a small aneurysm was seen at the beginning of the basilar artery, which was poorly visualized. The left internal carotid artery traffic segment was seen to be locally thickened, and the stump of the internal carotid artery was considered. The rest of the intracranial vessels were not significantly abnormal. Combining the patient's symptoms, signs, and ancillary examinations, the right vertebral artery aneurysm, a micro-aneurysm at the beginning of the basilar artery and bilateral common carotid artery occlusion were confirmed by imaging. The 8 F guiding catheter was then delivered to the V1 segment of the right vertebral artery under the guidance of a guidewire, followed by a 5F Navien intermediate catheter along the 8F guiding catheter to the V2 segment of the vertebral artery under the guidance of a microguide, fixing the 5F Navien catheter (Figure 3) and introducing the microguide and spring-coil catheter discreetly into the aneurysm under the guidance of Roadmap. The lumen was confirmed by imaging, and the Axium spring coil 6 mm ∗ 20 cm was slowly released into a basket, followed by the Axium spring coil 5 mm ∗ 15 cm 3D, Axium spring coil 4 mm ∗ 12 cm 3D, Axium prime spring coil 3 mm ∗ 8 cm 3D, and Axium prime spring coil 3 mm ∗ 8 cm 3D. A total of 6 spring coils were successfully implanted into the aneurysm cavity, and a relatively dense embolization of the aneurysm was seen on imaging from which the filling rate was calculated to be about 28%, with good visualization of the branches (Figures 4(a)–4(d)). Raymond's grade is grade 1. For the small aneurysm at the beginning of the basilar artery, the tumor body is small and the interventional operation is difficult. It can be rechecked regularly, so the operation was ended. After the operation, the arterial sheath was removed and the puncture site was compressed with a compression bandage.

## 4. Results and Observations

Postoperatively, the patient was given symptomatic supportive treatment such as blood pressure control, nerve nutrition, epilepsy prevention, vasospasm prevention, and intravenous nutrition. The patient was also given multiple lumbar punctures for replacement of blood cerebrospinal fluid. After treatment, the patient was discharged with a satisfactory recovery and a GOS score of 5 at one month postoperative follow-up observation.

## 5. Discussion

The common carotid artery has two terminal branches, which divide into the internal carotid artery at the level of the thyroid cartilage and the external carotid artery. In patients with bilateral occlusion or severe stenosis of the common carotid artery, the haemodynamic disturbances are often severe due to impaired cerebral blood flow autoregulation mechanisms and inadequate compensation of collateral vessels [5]. It has been shown that, as the degree of common carotid artery stenosis increases, the number of collateral circulation openings increases and the greatest number of collateral branches occurs with occlusion. And the rate of cerebral stenosis, the patient's age, and the compensatory capacity of the collateral circulation are negatively correlated [6]. Factors influence the establishment of collateral circulation of cerebral blood supply and its assessment. In this case, when bilateral common carotid artery occlusion occurred, combined with a slender left vertebral artery, the right vertebral artery assumed the main blood supply to the brain. The long-term haemodynamic changes increased the pressure of blood flow in the tortuous area of the vertebral artery, the basilar artery, and its branches and increased the risk of saccular aneurysm here. Some cases have been reported in which these aneurysms can be treated by craniotomy and have a good prognosis [7]. However, it has been suggested that the anatomical location of the aneurysm in close proximity to important neurovascular structures makes surgical access difficult. Secondly, because the anterior circulation has been compromised and the vertebrobasilar system is the only source of blood supply, the use of temporary clip block for proximal control is prone to serious complications due to the absence of intracranial compensatory vessels. Thirdly, because of the high intracranial pressure in the vertebrobasilar system, clamping of such aneurysms is likely to lead to intraoperative re-rupture and haemorrhage [8]. Meanwhile, Konishi et al. [2] reported a case of bilateral internal carotid artery occlusion combined with multiple intracranial aneurysms, which was successfully treated by craniotomy combined with endovascular embolization. Endovascular intervention has the characteristics of minimal injury and accurate localization and has been favored by many neurosurgeons and patients in recent years. Meguro et al. [9] reported a case of bilateral common carotid artery occlusion combined with endovascular stent-assisted coil embolization of an aneurysm of the bifurcation of the basilar artery and posterior cerebral artery by a double balloon remodelling technique. Kim et al. [10] reported a case of a male patient with a family history of Moyamoya disease who had a complete occlusion of the internal carotid arteries bilaterally combined with a ruptured aneurysm of the bifurcation of the basilar artery, which was eventually cured by endovascular spring coil embolization. Sameš et al. [11] reported a case of bilateral occlusion of the internal carotid artery combined with an aneurysm at the junction of the posterior communicating artery and the P1 segment of the posterior cerebral artery. Araki et al. [12] reported a saccular aneurysm at the junction of the right posterior cerebral artery with the right posterior communicating artery and one each at the P2 segment of the right posterior cerebral artery in a bilateral common carotid artery occlusion. Because of the high flow pressure in the vertebrobasilar artery and the fact that it is the main blood supply artery to the brain, compensating for almost all of the intracranial blood supply, it makes the treatment of aneurysms occurring in the posterior circulation branches more difficult and risky. Bilateral common carotid artery occlusion can occur for a number of reasons, such as atherosclerosis, aortitis, periarterial inflammatory lesions, vascular myofibrillar dysplasia, arterial entrapment, and radiation therapy injury [1, 13–15]. The most common of these is due to atherosclerosis, with more typical images. Atherosclerosis occurs at the beginning of the internal carotid artery and leads to a chronic progressive stenosis. When completely occluded, the stump of the artery has a “beak” shape on DSA, which is not easily detected clinically because it progresses slowly [16–18]. In addition to atherosclerosis, aortitis can also cause occlusion of the carotid arteries, and patients have a clear family history. Aortitis occurs in oriental women and most often involves the aortic arch and its branches, which leads to occlusion of the common carotid arteries bilaterally and ultimately to the absence of blood flow through the internal carotid arteries. In recent years, several studies have shown a genetic association with the development of vasculitis [19–21]. The absence of blood flow in the internal carotid arteries following occlusion of the common carotid arteries due to arteritis may have been the main cause of the bilateral occlusion in this case, with the same clinical outcome as the occlusion of the beginning of the internal carotid arteries due to atherosclerosis [22, 23]. However, the patient was negative for P-ANCA, C-ANCA, ANCA-MPO, ANCA-PR3, and ACA by relevant laboratory antibodies, although some studies have demonstrated that the relevant immunological markers may be negative if the aortitis is in a nonacute phase, and based on the patient's family history and angiographic findings, the possibility of bilateral common carotid artery occlusion due to aortitis cannot be excluded [24]. Due to the different pathological processes of atherosclerosis and aortitis, there are significant differences in DSA images. When bilateral occlusion of the beginning of the internal carotid artery is seen on DSA, atherosclerosis should be considered first, and when bilateral common carotid artery occlusion is seen on DSA, aortitis should be considered as a priority [1]. Certainly, cervical vascular occlusion may also be associated with other diseases, Fukaya et al. [25] reported a giant aneurysm of the posterior cerebral artery associated with bilateral internal carotid artery occlusion in a patient with Klippel–Trenaunay syndrome. Bilateral occlusion of the internal and common carotid arteries is mostly a chronic pathological process, which not only gives the posterior circulation time to adequately compensate for the whole cerebral blood flow but also some collateral circulation will gradually open or form to supply the occluded internal and common carotid arteries so that the intracranial blood supply will also reach a new equilibrium, but these gradually formed and opened collateral circulations mostly vary according to the location of the occlusion of the carotid arteries [26, 27]. The right vertebral artery, which had been supported for many years, was still overwhelmed due to haemodynamic factors, and the right vertebral artery V4 segment aneurysm ruptured and blew, along with a small aneurysm at the beginning of the basilar artery. These aneurysms can be treated with endovascular interventions and, if treated appropriately, can be treated satisfactorily.

## 6. Conclusion

A case of bilateral common carotid artery blockage and aneurysm in the V4 segment of the right vertebral artery with left vertebral artery constriction is described in this study. An elderly female patient with subarachnoid haemorrhage (SAH) was diagnosed with a V4 segment of right vertebral artery aneurysm, a microaneurysm at the beginning of basilar aneurysms, bilateral common carotid artery occlusion, and a narrowing vessel of left vertebral artery, thanks to improved digital subtraction angiography (DSA). In this case, endovascular treatment of bilateral common carotid artery occlusion and V4 section of right vertebral artery aneurysm resulted in outstanding clinical results. Although long-term follow-up is required, endovascular treatment of a bilateral common carotid artery occlusion associated with a V4 segment of a right vertebral artery aneurysm resulted in excellent clinical results in this patient.

## Figures and Tables

**Figure 1:** In Figure (a), the 5F Pigtail catheter was guided by a guide wire to the aortic arch. Bilateral common carotid artery occlusion was seen, the left vertebral artery was slender and poorly visualized, and the right vertebral artery was significantly thickened.

**Figure 2:** Figure (a) is anteroposterior view; a narrow carotid aneurysm with a neck of approximately 2.2 mm and a body of approximately 7.9 mm ∗ 7.5 mm is seen in the V4 segment of the vertebral artery on the right side of the figure.

**Figure 3:** (a) Anteroposterior view. (b) Left and right view showing the 8F guiding catheter and 5F Navien intermediate catheter climbing under guide wire guidance. (c) Left 45° view showing the 8F guiding catheter being delivered to the V1 segment of the right vertebral artery under guide wire guidance, followed by the 5F Navien intermediate catheter along the 8F guiding catheter under microguide guidance to the The 5F Navien catheter was then delivered along the 8F guiding catheter to the V2 segment of the vertebral artery under the guidance of a microguide wire.

**Figure 4:** The microguiding wire and spring-coil catheter were introduced discreetly into the lumen of the aneurysm under Roadmap guidance, and a total of six spring coils were inserted after angiographic confirmation (a) Magnified anterior-posterior view, (b) magnified left-right view, (c) magnified anterior-posterior view of the whole brain, and (b) magnified left-right view of the whole brain. Angiography showed that the aneurysm was relatively dense and embolized, and the vessels of each branch were well developed.

## Data Availability

The data used to support the findings of this study are included within the article.
